The article "The Application of Targeted Nanodrugs with Dual Responsiveness of PH and Ros in Preventing and Treating Vascular Restenosis" was retracted in 2023. Reasons: suspected computer-generated content; unreliable results or conclusions; concerns about the data; concerns about the results or conclusions.

# The Application of Targeted Nanodrugs with Dual Responsiveness of PH and Ros in Preventing and Treating Vascular Restenosis

**DOI:** 10.1155/2021/3982158

**Published:** 2021-11-26

**Authors:** Jin Zhang

**Affiliations:** North China University of Science and Technology Affiliated Hospital, Tangshan, Hebei 063000, China

## Abstract

In order to study the application of PH- and Ros-responsive targeted nanodrugs in preventing and treating vascular restenosis, a method based on pH-responsive and reactive oxygen species- (ROS-) responsive carrier materials synthesized in the early stage and rapamycin as a model drug was proposed. This method evaluated the therapeutic advantages of PH and Ros dual-responsive nanoparticles and the effect of dual-responsive active targeted drug delivery nanoparticles on vascular restenosis in vivo by comparing with nonresponsive PH or Ros single responsive nanotherapy. By optimizing the feed mass ratio of pH-responsive materials (ACD) and ROS-responsive materials (OCD), the best pH and ROS responsive nanoparticles were prepared. It has been proved that nanoparticles have ultrasmall volume (10–1000 nm) and can easily pass through the blood vessel wall without causing damage and have the characteristics of targeting and sustained release, so they are an ideal carrier for local administration. Nanoparticles as gene vectors have also achieved good results.

## 1. Introduction

In recent years, targeted drug delivery based on nanoparticles has been considered as a promising strategy for specific delivery of different imaging and therapeutic drugs, providing a new approach for the diagnosis and treatment of cancer and immune, cardiovascular, and other diseases. Cardiovascular disease (CVD) is the main cause of morbidity and mortality in the world. It is estimated that cardiovascular diseases can cause 17.9 million deaths every year, accounting for about 31% of the total global deaths. Studies have shown that vascular inflammation is closely related to the pathogenesis of many cardiovascular diseases, such as atherosclerosis, myocardial infarction, restenosis, intracranial aneurysm and aortic aneurysm, stroke, and peripheral artery disease. By regulating different molecular and cellular processes involved in inflammatory reactions, a large number of therapeutic methods have been studied to prevent and treat cardiovascular diseases [1]. Although great achievements have been made in preclinical research, however, the ideal efficacy of most tested anti-inflammatory drugs has not been fully proved in clinical practice. To a great extent, this may be related to the inefficient delivery of therapeutic molecules to vascular inflammation sites, which is caused by their nonspecific distribution and rapid elimination from circulation. Even drugs are absorbed locally in inflammatory blood vessels because of uncontrolled diffusion, and the residence time is also very short. In recent years, targeted therapy based on nanoparticles is considered as a promising strategy, which can specifically deliver different therapeutic and imaging drugs for detecting or treating vascular inflammation [2]. Especially, a wide range of nanoparticles have been designed as targeted carriers to treat atherosclerosis, myocardial infarction, heart failure, ischemia-reperfusion injury, severe limb ischemia, restenosis, abdominal aortic aneurysm, and ischemic stroke. In these examples, polymerized lipid nanoparticles, liposomes, recombinant high-density lipoproteins, vesicles derived from cells, inorganic nanoparticles, metal nanoparticles, and mixed nanoparticles are used to deliver therapeutic drugs [3]. In addition to passively targeting vascular lesions through a damaged endothelial cell layer or EPR effect, nanoparticles can further improve vascular targeting efficiency by adjusting their physical properties (such as geometric structure and compliance), modifying molecular groups, or functionalizing special cell membranes. Studies have shown that according to the biochemical signals of abnormal changes of vascular inflammation sites, people can design and synthesize the components of nanoparticles and release the drug load in a targeted manner. However, the transformation of these vascular targeted nanotherapies is still challenging [4]. Siracuse J. et al. believe that although direct regulation of antigen-specific affinity can enhance the aggregation of nanoparticles in blood vessels, the targeting efficiency of nanoparticles is still very limited only after modification with molecular groups. For nanodrug therapy derived from the biomimetic strategy based on cell membrane, its relatively complex formulation process and unclear components may hinder its subsequent large-scale production and clinical research [5]. Cf A. thought that, in view of the slight acidic environment of inflammation and increased oxidative stress after vascular endothelial injury, active oxygen and pH-responsive nanoparticles were constructed by integrating and optimizing the ratio of active oxygen and pH-responsive cyclodextrin materials, which can be used as a new effective and safe nanoplatform for drug delivery at vascular inflammatory sites [6].

## 2. Treatment of Vascular Restenosis

According to the characteristics of vascular restenosis, researchers have put forward some treatment schemes to inhibit vascular restenosis, but there is no completely successful treatment method in clinic.

Because systemic therapy cannot successfully inhibit restenosis, researchers put forward the concept of local administration. The main advantage of local administration is that the dosage is reduced, thus alleviating the toxic and side effects of drugs, and the local action time can be prolonged through the physical or chemical connection between drugs and carriers. In addition, short-half-life drugs, such as recombinant proteins, polypeptides, and other unstable biological macromolecules, can reduce the damage caused by systemic administration. Local administration can also avoid individual differences [6–9]. Therefore, from a therapeutic perspective, the development of drug vectors that can effectively deliver bioactive agents and selectively target regions of oxidative stress and acidic microenvironment may play a positive role in the diagnosis and treatment of inflammation-related diseases.

### 2.1. Peripheral Administration of Blood Vessels

The principle of peripheral administration of blood vessels is to provide a drug reservoir on the outer skin of blood vessels, from which the drug is released into tissue fluid and passively diffused into the blood vessel wall driven by concentration gradient. Ethylene-vinyl acetate copolymer (EVA) is a nontoxic biodegradable polymer. It has been approved by the FDA as a carrier for peripheral drug delivery. It can carry lipophilic or hydrophilic drugs and has good mechanical properties. Researchers systematically studied the antiproliferation and restenosis effects of heparin carried by EVA in the rat carotid artery model. Experiments show that local extravascular administration of heparin is an effective method to prevent restenosis. EVA can also carry antisense oligonucleotides as a vector [6].

### 2.2. Intravascular Administration

Intracavitary administration can be performed simultaneously with percutaneous vascular intervention. Once administered, the drug is first distributed in the deepest part of the intima and middle layer of blood vessels, so it can treat intravascular processes such as thrombosis. Then, some drugs were redistributed through the vascular nourishing tube and reached the adventitia. Because redistribution is performed in a few hours, treatment can occur in the process of adventitia, such as the aggregation of myofibroblasts and the change of connective tissue protein expression [10].

### 2.3. Intraluminal Stent

In recent years, with the in-depth study of vascular deformation after interventional angioplasty, endovascular stents have been widely used. The mechanical force of stent can neutralize the early elastic recovery of blood vessels and the late contraction deformation of blood vessels, but the intimal hyperplasia caused by stent is more serious than that caused by interventional angioplasty. In order to prevent restenosis caused by stent, researchers have proposed two new drug delivery systems based on stents. One is to wrap a polymer film containing drugs on the stent. The other is made of biodegradable polymer containing drugs [11, 12].

Commonly used vectors for gene therapy of vascular restenosis mainly include adenovirus vector, retrovirus vector, liposome, cationic polymer, etc. Adenovirus vector is the most widely used gene vector at present. Adenovirus transfection efficiency is very high, and it will not integrate into the DNA of host cells, so there is no risk of carcinogenesis. There are some problems in the use of viral vectors in gene therapy, such as their immunogenicity, proto-oncogene characteristics, and some unknown long-term effects. Nonviral vectors do not have these problems. However, the transfection efficiency of such vectors as liposomes is relatively low. The transfection efficiency of cationic polymer is relatively high, but its clinical applicability needs further research. Stimulus-responsive nanoparticles have been widely concerned as an intelligent drug delivery system and used in the diagnosis and treatment of various diseases.

## 3. Application of 3 Nanoparticles in the Treatment of Vascular Restenosis

Nanoparticles are new drug controlled-release carriers made of polymer with a diameter of 10–1000 nm. Drugs can be wrapped inside nanoparticles or adsorbed on the surface of nanoparticles, or they can be combined with nanoparticles through chemical bonding. Nanoparticles can carry different drugs [13], and their release time ranges from several minutes to several months. The mechanism of drug release from nanoparticles can be drug diffusion, polymer degradation, or adsorbed drug detachment from nanoparticles.

As a drug delivery system, nanoparticles have certain advantages for local drug delivery in blood vessels. Because of its very small volume, it can easily pass through the blood vessel wall. It can easily enter the blood vessel wall without causing damage. According to the different physical and chemical properties of drugs, the drug loading of nanoparticles can reach up to 30%. By adjusting the parameters of the preparation process and the composition of the polymer, the release time of the coated drug can be from several days to several months. Nanoparticles can be made into uniform and stable suspension and dispersed in salt solution or buffer solution and can also exist in tissue culture solution. Therefore, it is feasible for injection. In addition, due to the small size of nanoparticles, when it enters the body, it hardly causes the immune response of the body. Studies on the distribution of viscera confirmed that the distribution of dual-responsive nanoparticles in vivo was mainly concentrated in the liver and spleen, relatively less in the lungs, and almost no fluorescence distribution in the heart and kidney after injection of the tail vein.

Studies have shown that local administration of dexamethasone nanoparticles coated with poly (lactic acid-polyglycolic acid) copolymer can effectively inhibit restenosis in rat carotid artery and pig coronary artery models [3], and dexamethasone has existed in blood vessel walls for more than two weeks. U-86983 (an antiproliferative agent) nanoparticles have an obvious antiproliferative effect in tissue culture, and continuous application in the rat model for two weeks can inhibit the occurrence of restenosis. Heparin-loaded poly (lactic acid-polyglycolic acid) copolymer nanoparticles can reduce platelet deposition by nearly 40 times in the pig vascular model, and the coagulation time has not changed, which indicates that heparin does not show a systemic effect. Therefore, local administration of heparin nanoparticles can effectively inhibit thrombosis and restenosis of blood vessels [1] and, at the same time, lead to endothelial dysfunction, macrophage activation, and release of cytokines and growth factors, promote the proliferation and migration of vascular smooth muscle cells, and ultimately, lead to the formation of new intima and lumen stenosis.

## 4. Experimental Analyses

### 4.1. Materials and Methods

In this experiment, PLGA nanoparticles containing RPM were prepared by ultrasonic reemulsification and solvent evaporation. RPM is added into methylene chloride solution of PLEA with a certain concentration and volume, and ultrasonic emulsification is carried out by using a probe ultrasonic instrument under ice bath condition to form a uniform suspension, then PVA aqueous solution is added, and stirring is continued by the ultrasonic emulsification instrument to prepare a uniform milk-like compound emulsion. It is put in a beaker, and the organic solvent is volatilized with a magnetic stirrer at normal pressure in a fume hood. After the solvent is completely volatilized, it is centrifuged with a high-speed centrifuge at 23000RPM for 20 minutes and the supernatant is discarded. The collected precipitate is washed with distilled water for 3 times and then freeze-dried for preservation after removing free rpm and PVA. The level of H_2_O_2_ was significantly reduced after treatment with double-responsive rap-loaded nanoparticles, indicating that the double-responsive rap-loaded nanoparticles can effectively reduce the oxidative stress of damaged local tissues. The process flow is shown in Figure 1.

The animals were killed by euthanasia at 1 hour and 3 hours after operation, the hearts were taken out quickly, and the coronary arteries were washed with normal saline. The administration position was determined with reference to CAG, and the administration vessel was dissociated. A total of 4 cm blood vessels were taken from the 1 cm above and below the estimated position in the drug administration group, and 2 cm blood vessels from the dyeing position in the dye group were placed in an Eppendorf tube for marking and then stored in a liquid nitrogen tank. The blood concentration sample is cut in time. Tissue homogenate was performed in a tissue homogenizer. After centrifugation, the supernatant was taken and stored at low temperature [14].

RPM detection conditions by HPLC are shown in Table 1. RPM content of the arterial wall was measured by an internal standard method and external standard method, respectively.

Pretreatment before injection: the sample was dissolved by 0.5 *ml* mobile phase and centrifuged at 10000 rpm for 3 min, and 50 *μl* sample solution was absorbed and injected.

### 4.2. Selection of Internal Standard

N, N-diethyl-m-toluamide (deft) was selected as the internal standard for detecting RPM by HPLC. Internal standard retention time after injection shall be interpreted with reference to the injection time of separate internal standard.

1. Selecting an internal standard method for drug extraction in vascular tissue
2. Taking out the vascular tissue from the Eppendorf tube and accurately weighing the wet weight of the tissue
3. Cutting the tissue pieces evenly and putting them into a tissue homogenizer and adding 50 *μl* internal standard solution, 1 *ml* homogenizing normal saline, and a proper amount of rapamycin standard solution
4. Taking the suspension and adding it into the centrifuge tube and addding chloroform solution 1 *ml* at the same time, then oscillating for 15 min, and centrifuging at 3000 rpm for 10 min
5. Absorbing the lower organic phase and putting it in a clean test tube
6. 1 *ml* chloroform is added into the upper water phase again. The abovementioned steps are repeated, and the organic phase is added into the storage test tube
7. Storing the test tube of organic phase in an oven at 500C overnight and draining it the next day
8. The mobile phase was added to the sample for HPLC detection [15]
9. The external standard method is the same as the internal standard method except that the internal standard solution is not added in the step
10. Testing the standard curve and reproducibility
11. Taking 6 abdominal aorta of New Zealand white rabbits with a diameter of about 2.5 mm and a length of about 40 mm and accurately weighing the wet weight of the tissues
12. Cutting the tissue block evenly, putting it into a tissue homogenizer, and adding l1 ml normal saline and a proper amount of rapamycin standard solution for homogenization

The recovery rate was determined, and the RPM concentrations were 6.25, 25, and 50 *μg*/*ml* for each standard solution. 1 *ml* 6.25, 25, and 50 *μg*/*ml* standard solutions are added into the cut arterial tissue, extracted according to the abovementioned conditions and methods, and measured by HPLC, and 20 *μl* samples are injected each time, and each concentration was determined 4 times repeatedly. 1 *ml* 2.5 *μg*/*ml* RPM standard solution is added into the cut arterial tissue, extracted according to the abovementioned conditions and methods, and measured by HPLC, and 20 *μl* samples are injected each time, and the determination was repeated 5 times. At the same time, in the microenvironment of inflammation and oxidative stress at the site of vascular endothelial injury, pH and ROS dual-responsive drug-loading nanoparticles can simultaneously trigger the release of the drug rapamycin in the slightly acidic local tissues and the elevated ROS environment and inhibit the proliferation and migration of VSMCs, thus more effectively inhibiting the formation of angiogenesis intima.

### 4.3. Statistical Treatment

All data were calculated by SPSS10.0. The statistical results are expressed as mean and standard deviation (measurement data) or percentage (counting data). The data were tested for normality by the Kolmogorov–Smirnov method. The parameters among groups in the normal population were compared by the *T* test or Newman–Keuls test of one-way square analysis. Rank and Kruskal–Wallis tests were used for nonnormal distribution data. The *X* test and Fisher accurate probability test were used for counting data. Confidence coefficient was taken as *α*=0.05.

## 5. Results

The particle size distribution of RPM-PLGA nanoparticles prepared by ultrasonic emulsification can be seen from the light scattering particle size distribution diagram. RPM-PLGA nanoparticles prepared by PLGA with an LA : GA ratio of 50 : 50 have an average particle size of 246.8 nm, and the particle size distribution is concentrated in the range of 208nm-294 nm, showing a narrow distribution [16].

The sample of RPM-PLGA nanoparticles prepared by ultrasonic emulsification was observed by using a scanning electron microscope, as shown in Figure 2. Nanoparticles are spherical, smooth in appearance, and well encapsulated. It can be seen that the particle size observed by using the SEM is within the expected range, which is consistent with the light scattering results. The flaky lump shadow can be seen in the photo because the HITACHIX-650 scanning electron microscope cannot cool the sample at the same time, and the high temperature under the microscope melts the RPM-PLGA nanoparticle sample. We intend to further construct dual-responsive nanodrugs targeting intravascular subcutaneous type IV collagen by modifying pH and ROS dual-responsive nanoparticles with targeting units and characterize their physical and chemical properties.

The free RPM-PLGA was extracted according to the abovementioned method, and the experimental results showed that the average extraction rate reached more than 99% (Table 2), so the reliability of this method for determining the drug embedding rate of RPM-PLGA nanoparticles can be affirmed.

The research shows that type IV collagen (Col-IV) is the main component of subcutaneous basement membrane in blood vessels, and KLWVLPKGGGC polypeptide has high affinity with type IV collagen and has good targeting for inflammatory and/or injured vascular lesions. In view of the abovementioned situation, we covalently bound the polypeptide with DSPE-PEG-maleimide by chemically bonding sulfhydryl with maleimide. DSPE-PEG-KLWVLPKGGGC was successfully synthesized, and then, TAOCD NP (pH/ROS Double-Responsive Nanoparticle) targeting intravascular subcutaneous type IV collagen was successfully prepared by a similar nanoprecipitation/self-assembly method. TEM and SEM observations show that TAOCDNP is spherical, with uniform particle size and good dispersion. Compared with the RAP/AOCD NP treatment group, the RAP/TAOCD NP treatment group was more effective in increasing the lumen area, reducing the new intima area, and decreasing the arterial proliferation index.

In this study, pH/ROS biresponse IV nanoparticles (TAOCD NPs) targeting intravascular subcutaneous collagen type IV were successfully constructed by a similar improved nanoprecipitation/self-assembly method. The antiproliferative drug RAP can be effectively encapsulated into TAOCD NPs to form a targeted and double-responsive drug-loaded nanoparticle (RAP/TAOCD NP). In vitro studies show that similar to nontargeted nanoparticles (AOCD NPs), Cy5/TAOCD NPs can be effectively absorbed by rVSMCs in a dose-dependent and time-dependent manner. Cy7.5/TAOCD NPs can specifically bind to type IV collagen in vitro. After being modified by targeted type IV collagen polypeptide, the biresponsive nanoparticles significantly enhanced their ability of targeted aggregation of injured carotid artery tissue. The dual-responsiveness-targeted RAP nanoparticles significantly inhibited the abnormal proliferation of neovascular intima after balloon injury of the carotid artery in rats and further improved the effect of pH/ROS dual-responsiveness nanodrug in preventing and treating vascular restenosis in vivo. Cy7. 5/TAOCD NPs can specifically bind to type IV collagen in vitro. Dual-responsive nanoparticles modified with targeted type IV collagen peptides significantly enhanced their ability to target aggregation of injured carotid artery tissue.

## 6. Conclusions

Based on the abovementioned research results, we believe that the pH of constructing based on beta-cyclodextrins and the ROS double-responsiveness nanodrug delivery system can effectively deal with the active species with low pH value and high level caused by endothelial injury and effectively release the drug carrying molecules in the environment of microacid and oxidative stress, so as to avoid systemic toxicity to the drug. Moreover, the targeting ability of AOCD NPs was significantly improved by modifying the targeting unit of the double-responsive nanocarriers. From what has been discussed above, we can see that the nanoparticles with ultrasmall volume and high drug-polymer interactions can easily penetrate the vascular wall instead of the vascular endothelial damage and also can reduce the side effects of drugs, protect the drug from enzymatic degradation, and so on, so the nanoparticles in the treatment of vascular restenosis have a unique advantage. However, there are also some problems in the application of nanoparticles, such as the biocompatibility and biodegradability of materials, the stability and integrity of biological macromolecules carried by nanoparticles, and the content and release time of drugs in nanoparticles, and all need to be carefully investigated. Therefore, we can imagine that using nanoparticles as gene carriers for gene therapy is a promising research direction [17].

## Figures and Tables

**Figure 1:** Schematic diagram of preparation of 1RPM nanoparticles.

**Figure 2:** RPM-PLGA nanoparticle size distribution diagram.

**Table 1:** Conditions for detecting RPM by HPLC.

RPM conditions were detected by HPLC	
The chromatographic column	C18250^*∗*^4 mm
Mobile phase	65 : 35
The velocity	1.0 ml/min
Ultraviolet detection wavelength	277 nm
Retention time	9.0 min

**Table 2:** Free RPM-PLGA extraction results.

Group	RPM extraction amount (mg)	The RPM the inputs	The extraction rate (%)	Average extraction rate (%)
1	2.854	3.01	94.817	96.347 + 1.326
2	2.954	3.04	97.171	
3	2.931	3.02	97.053	

## Data Availability

The data used to support the findings of this study are available from the corresponding author upon request.
